# Analysis of Ecological Environment Problems and Countermeasures in Ideological and Political Education in Colleges and Universities

**DOI:** 10.1155/2022/9479881

**Published:** 2022-10-12

**Authors:** He Hao

**Affiliations:** Jilin Police College, Changchun City, Jilin Province 130017, China

## Abstract

At present, there are many problems in the mode and method of ideological and emotional education of college students. The state attaches great importance to this aspect and continues to increase investment, but the effect is not satisfactory. As an important field for cultivating high-level socialist talents, colleges and universities have played a huge role in promoting the ideological development and emotional education of college students. The emergence of this contradiction shows that traditional educational methods have their own shortcomings and need to expand their thinking and explore new research areas. Since the new era, the ideological education venues and teaching activities of colleges and universities have been greatly improved, but they are also facing many problems and challenges, which seriously affect the moral quality of college students and destroy the ideological education ecosystem of colleges and universities. From the perspective of the ecological crisis of education, this paper awakens and pays attention to the ecological problems of education, making it an inevitable trend of current education development and paving the way for future research. On this basis, the current situation of the ecology of political education of college students is analyzed, and the necessity of research is proposed. Analyzing the ideological and emotional education of college students from the perspective of ecology is essentially to regard the ideological education of college students as an ecosystem and deeply analyze the distribution of various components and elements of college students' ideological and political education. The ecology of college students' ideological education is the process, law, and overall ecological balance of various factors in the ideological education system of college students, as well as the methodological thinking and value orientation of the interaction between various factors and the environment. The changes of the ecological environment have a significant impact on people's state of mind. As college students growing up in the new environment, their thoughts, emotions, and values are all affected by the development of the ecological environment. Therefore, changes in the ecological environment, air quality, and water environment have increasingly obvious impacts on the living environment.

## 1. Introduction

### 1.1. Ecological Connotation of Classroom

State system refers to the combination of life subject and surrounding environment in a certain space. The same is true of classroom ecology, which is embodied in classroom space and the relationship between biology and environment. Doyle and Pound point out that “the context of every learning activity includes the student, the teacher, the background and the learning information, so learning takes place in an ecosystem.” In this system, the interaction and positive influence of various factors form a unique classroom ecosystem (see Figure 1).

As a whole, teachers and students are in the ecosystem of the classroom [1]. This sentence has two meanings: one is the interactive relationship between teachers and students in the classroom ecological environment. The living state and development trend of classroom ecological subject are maintained and changed in various ways. They depend on each other and influence each other, constituting a whole classroom ecosystem. The second is the mutual reference between teachers and students, forming two different classroom ecological subjects: teachers' ecological groups and students' lives. Teachers take students as reference in the teacher group and form a teacher ecosphere among themselves. There are a variety of formal or informal spiritual or material relations between teachers and groups. Under the guidance of teachers, students form a student ecosystem, which also includes individuals. Different relationships between groups in the progress of education information management was studied [2]. The relationship between the two is complex. They influence each other. They are interrelated. Classroom ecology is a unique ecosystem with integrity, openness, symbiosis, and balance.

First of all, classroom ecology is a whole. From the point of view of systems, an ecosystem is a real, not illusory, existence. The totality of nature is a higher organization than its own organic members, presenting beauty, stability, and integrity. It is a way of life. Secondly, the ecological environment of the classroom is open. Betalangfei, the founder of the generalized system theory, believed that the organism is an open system; that is to say, all organisms must survive under appropriate conditions and must be open; that is to say, only by constantly communicating with external matter, energy, and information can they survive. Symbiosis is a common characteristic in the evolution of organisms and an important link between organisms. Finally, the classroom ecosystem is balanced. From the perspective of ecology, ecological balance refers to the relative stability of the structure, function, material energy, and information input and output of an ecosystem.

### 1.2. Analysis of Basic Concepts of Ecology and Environment

In different backgrounds, people's understanding of ecology and environment is different. In biology, the term “living body” refers to “an organism and its surrounding structures that exhibit an association of energy (energy flow, matter flow, information flow).” In this system, there are many branching structures in the analysis of functional relationships [3]. In ideological education, “ecology” refers to the survival and development of students under specific natural conditions. Sustainable development of education. Environment refers to the space in which human beings live and various natural factors which can directly or indirectly affect human life and development. In this process, students are the main body; emphasis on the main body helps them become people-oriented, pay attention to humanistic care, and embody more the ecological benefits of ideological and political education.

### 1.3. Research on the Historical Background of Ecological Civilization Education

“Ecological civilization” raises the issue of “humans” to a new level, with higher requirements for “humans,” which requires the all-around development of “humans,” “all-around” promotion of “humans,” and being “people-oriented.” The formation of ecological civilization is closely related to people's bad behavior [4]. As shown in Figure 2, the emergence of ecological and environmental problems is the product of multiple factors. First, the rapid development of industrial civilization has greatly improved the level of industrial automation but also brought a lot of sewage and waste gas. Sewage discharge will not only pollute the environment but also cause certain damage to the natural inherent ecosystem, causing great damage to the ecological environment, and making it impossible to recover. People depend on the natural environment to live; we should protect the ecological environment and create a beautiful landscape. Second, human beings continue to plunder nature, resulting in a sharp decline in natural resources. The large-scale and unplanned exploitation of human resources leads to the exhaustion of various mineral resources, which leads to the frequent occurrence of various ecological disasters. We should set up the correct concept of interest and value, safeguard the ecological environment, and promote its healthy development. Third, the ecological carrying capacity has reached its limit. The carrying capacity of nature is limited; it must be in a relative balance; otherwise, it will endanger the survival and development of human beings. The frequent occurrence of natural disasters beyond the natural carrying capacity poses a great threat to human existence. College students should consciously realize the ecological concept of harmony between man and nature and realize the balance of all kinds of relations in nature, so as to realize the harmony of the biological world and thus form a new ecological concept.

### 1.4. Think about the Status of Education

The ecology of ideological education refers to the educational object around which the concept of ideological education is centered. Only on the basis of understanding this, can we prepare for the follow-up research. Some people believe that the ideological education environment is the objective reality that ideological education is surrounded by and affects the object of education. Some people put forward that it is the sum of all external factors that affect the formation and development of people's ideological and moral character and affect the operation of ideological education activities. Here is a typical point of view that many scholars have a consensus; different scholars may be slightly different in language expression, but it is always discussed that the influence of an external objective reality on people and ideological education and the dialectical relationship between ideological education environment and education object are standing in opposition. Domestic scholars hold different views on the ecological understanding of ideological education [5]. Some people think that “ecological ideological education refers to the use of ecological principles and methods to think about ideological education, thinking education as a system of state, a comprehensive analysis of the relationship between the internal and external elements of the system, to improve the effectiveness of thinking education to make it systematic, harmonious and sustainable development.” Some others put forward that “based on the law of the development of thinking education and education, we should guide the work of thinking education and education in colleges and universities by the point of view of thinking, and optimize its structure with the help of the principle of thinking and method to promote the teaching and education of thinking and self. The harmonious development of nature and society shows the dynamic balance of the ideological education system.”

## 2. Description of the Problem

### 2.1. The Fault between Ideological Education System and Ecological Environment in Colleges and Universities

The ecological environment of college students' ideological education is its external condition [6]. It is the objective basis for the formation and development of a person's moral character. The environment content is complex and multidimensional; multi-ideological education is constantly changing people's thinking and behavior and affecting their work effect and process. As shown in Figure 3, the ecological environment of ideological education can be divided into “external” and “internal” categories. The external environment of the school has a certain influence on students' thoughts, while the internal educational environment is the teaching environment of the school. At present, China's education is facing a great challenge, that is, the conflict between the external environment and the internal environment. Externally, from the environment, colleges and universities and even the whole university are in a high level of variability.

In this transformational social environment, the transformation is reflected in the following: the status of the transformation to the whole society. Economic development is also the transition from planned economy to socialist market economy; in this environment, cultural industry will inevitably embark on the road of diversified development. This external environment is full of various information, which is also used for transmission. Accordingly, the teaching contents and teaching methods of the inner teaching circle are the same. The frequency of strengthening with the external environment compared to the speed means that the content of strengthening the internal environment is simply out of reach. If he does not respond, he will not only be completely defensive in the battle of ideas but also face “information overload.” No. The contradiction of the internal and external environmental factors is interwoven with the social and economic transformation, which easily makes the college students' lose self-control and the adjustment ability of thought, and then produce the dislocation of belief and life values, and then weaken its role.

At present, ideological work in colleges and universities is still a systematic project [7]. The ideological work of college students needs the support and cooperation from all aspects of family and society. Only by carrying out ideological work comprehensively can we create a good social environment and promote the physical and mental development of college students. But the truth is always disappointing [8]. First of all, due to the disconnection between family education and college education, some parents blindly pursue the intelligence and future of their children and neglect the moral education of their children. At the same time, due to the lack of communication between parents and schools, information exchange channels between schools and families are not smooth, which leads to the inability of family education and school education to form a joint force and promote the overall development of students. Secondly, due to the current social situation, especially the bad environment around the school, its role has been greatly weakened. In the transition period, the complexity and pluralism of social values, the bad social atmosphere and corruption, as well as the negative effects of western cultural trends have exerted an extremely negative influence on the overall development of college students, making social education deviate from its purpose.

### 2.2. Main Problems of Ecological Civilization Education in Ideological and Political Education in Colleges and Universities

#### 2.2.1. The Supply of Educational Methods Needs to Be Innovated

First, strengthen innovative teaching methods [9]. In ecological construction, the method of educating objects is not novel enough. In the case of ecological civilization teaching for “current ideological and political course” teachers, only 28.46% choose actual experience, while the rest are 67.23%, 60.46%, and 29.69%, as shown in Figure 4. Therefore, in ecological humanities, knowledge education is still the mainstream, focusing on the transmission of knowledge, but ignoring the actual participation. In the classroom, due to the limitation of time and space, it is difficult to combine the static, dynamic, and value needs of the human ecological environment with practical education and ability education. Due to the lack of ecological practice and students' environmental protection practice activities, the negative effects of environmental protection consciousness of college students are desalted and blurred, and it is difficult to have a profound and lasting impact on the cultivation of students' ecological quality.

Second, strengthen the educational methods for students [10]. In China's ecological construction, there exists a binary opposition of subjectivity and passive acceptance. The teaching method based on “teaching” has difficulty in breaking through the traditional teaching mode, ignoring the students' subjectivity and the disorder of thinking, thus affecting the subjectivity. Suhomlinsky believed that only through one's own efforts can one obtain and experience, which can be called true education. The self-education of S-level students is very important, which should move from heteronomy to self-discipline. A teacher's teaching is one, and thought is another. In the teaching process, teachers still remain in the sorting of the internal environment of education, so that students feel that teachers' teaching methods are not novel enough, their interest in the knowledge they have learned declines, and the learning effect is not good.

#### 2.2.2. The Supply of Educational Efficiency Needs to Be Improved

Ecological education plays an important role in the ideological education of college students [11]. However, from the actual performance, the problem of ecological environment deterioration is “on-site,” many ecological civilizations show that consciousness is an “empty field,” the subject consciousness is not strong, ecological awareness and executive ability are far from people's expectations, and the cultivation of green living habits has not been formed.

First, we do not fully understand ecological civilization. You need to obtain new information through various channels on the basis of professional ability, so as to improve their ecological civilization quality. The majority of students (59%) are case by case. A small number of them think it is not necessary, because as can be seen from the chart, most students do not take ecological civilization as an important factor to cultivate but as an auxiliary factor or even optional (see Figure 5).

Second, the study of ecological environment knowledge is not complete and comprehensive. What was the meeting about “the first time governments have come together to discuss a global environmental protection strategy”? Of the world's three major holidays, the correct answer for Earth Day is 29.6.9. As shown in Table 1, when asked about the grammatical meaning of “environment,” in terms of constructing “ecological” grammar and content, students are more inclined to choose “familiar” and “concise” under various circumstances where the “garbage classification” standard is strongly advocated, while less than 10% choose “very good.” It can be seen from this point that the current college students have not fully mastered the basic knowledge of ecological environment, some things taken for granted have not become real knowledge, and most of the knowledge is still at the most basic cognitive stage.

## 3. State of the Art

### 3.1. Current Situation of Ecological Civilization Construction of College Students

At present, the research on the construction of university ecological construction is not balanced enough, and the research focus is not prominent [12]. The paper points out that the current research on university ecological civilization is not comprehensive enough, and the attention to it is insufficient. As shown in Figure 6, at present, scholars at home and abroad have carried out a lot of discussions on ecological education for college students, but most of them lack practical significance and are difficult to apply in practice. Only in-depth discussion on its feasibility can effectively improve its teaching quality. Therefore, we must combine theory with practice and use theory to reveal problems, understand problems, solve problems, and actively solve environmental problems.

The research of ecological civilization education in foreign countries is earlier, and there are great innovations and achievements in methods. Environmental education was first developed in the West, and it was also the West that carried out environmental protection research and publicity, and achieved good results. Foreign countries have formulated environmental protection laws and regulations and carried out environmental protection propaganda in schools at all levels. In particular, in the United States, the characteristics of its environmental education is particularly prominent. In foreign countries, people have been strongly influenced by humanism. The transformation of anthropocentrism emphasizes the conquest and control of human beings over nature, which violates the operation law of nature to some extent, leading to the imbalance of ecological environment and serious ecological disasters and environmental problems.

### 3.2. The Significance of Classroom Ecology

From Confucius' “Apricot Terrace” to today's classroom, classroom has always been the main place for teachers and students to grow up and the inheritor of teachers and students. The quality of class ecological environment is directly related to the growth and success of students. God should proceed from the relationship between teachers and students, educational content, educational methods, and educational objectives.

#### 3.2.1. The Development of Classroom Ecology Has Promoted the Reunderstanding of the Relationship between Teachers and Students

The traditional connection between teachers and students is a challenge [13]. The theory of “one yuan” and “two subjects” is closely related to the traditional teacher-student relationship theory. In the ecological environment of the classroom, neither the teacher-centered student subject nor the teacher-centered student subject can reflect the ecological concept of harmony and equality. The emergence of the theory of “intersubjectivity” opens up a new era for the teacher-student relationship in the classroom ecosystem. The interaction between teachers and students is interactive, such as the exchange of information and feelings. In teaching, teachers should convey educational knowledge and ability to students with vivid expression, rich content, diversified teaching methods, and equal attitude.

#### 3.2.2. Promote the Rational Allocation of Teaching Content and the Ecological Construction of Classrooms [14]

The traditional task of classroom education is to transform knowledge into knowledge. It is reasonable for educators to teach it to the educated, including the quality-oriented education advocated today, but his original intention has not changed. The question, however, is how you should interpret what you are teaching, which goes against the text. The classroom ecological environment requires interaction between students. The transfer of information and the exchange of energy—that information should be healthy and beneficial and help maintain and contribute to the smooth functioning of the ecosystem. Therefore, if you want to achieve a virtuous circle, the most important thing is the dissemination of information. Fluency, that is, the arrangement of teaching content, should be reasonable; there should be goals. First of all, knowledge cannot be completely objectified, especially ideological and political work. Secondly, the connotation of knowledge should not be too narrow.

### 3.3. The Enrichment of Ideological and Political Education in Colleges and Universities by Ecological Environment

The components of ideological and political education activities include educational objectives, educational tasks and educational principles [15]. On the basis of modern education, modern education is not only the cause of full-time institutions such as schools but also the cause of the whole society. It may not only be relevant to everyone's childhood, adolescence, and youth period but may also be relevant to people's life, not only to make a living but also to live a better life and develop themselves better. The openness, trapezoid and flexibility of the school system; Modernization of education. The modernization of education includes the modernization of the educational system, objectives, concepts, contents, methods, means, teachers, facilities, and management. The goal of educational modernization is to cultivate modern people. Universality and immediacy of social connection, as well as the setting of teaching contents and methods, are influenced by a variety of environments. First, we must strengthen ideological and political work [16]. The educational thought, educational goal, and educational principle established by the educational subject are all summarized and refined to the provided educational materials [17]. Secondly, the influence of the subject of ideological education on the object of education is correct. Materials provided by the environment have been carefully selected. In the process of education, the ideas and data sources and object environment to be conveyed, that is, the educational content, are the result of the independent choice of material provided by the education object in the teaching situation. Third, the ideological education situation is a kind of educational situation deliberately created by the implementation subject. Literary scenery, various scenes designed by educators, and special atmosphere are all important contents of ideological education. The “educational platform” works on goals.

### 3.4. Ecological Man: An Important Symbol of the All-Around Development of Human Beings in the New Era

The ultimate goal of ecological construction is “people-oriented,” which has internal consistency with the overall development of human beings. At the same time, he is applying it to various societies and pushing it forward. The all-around development of human beings has the characteristics of the times, and its development emphasis has changed gradually in each historical stage. In the harmonious development of the relationship between man and nature, because the ecological needs of man have been put on the agenda, ecological construction must have a form suitable for the body. Therefore, in the new period, cultivating the value concept of “ecological man” with life rationality as the core is the need of the overall development of human beings. The all-around development of people is to constantly improve their physical fitness and constantly cultivate and develop their own abilities. This is not only to satisfy people's wishes but is also the foundation of a person, and he has an advantage over others. The goal of man's all-around development in the new era is not only to realize the “harmony” of man but also to realize the benign interaction and harmonious coexistence between man and nature. In this context, the ideological and political education of ecological civilization can help these children, who are the earliest to enter the ranks of “ecological people,” who will better promote the improvement of human comprehensive quality and all-around development, thus accelerating the process of ecology.

## 4. Result Analysis

### 4.1. Optimize the School Environment of Ecological Education for College Students

We should start from creating a good classroom teaching environment and strengthen the construction of campus ecological civilization. The construction of ecological culture is an important part of colleges and universities. We create excellent campus culture from three aspects. The advantages and disadvantages of ecological campus environment directly affect the effect of ecological civilization education of college students and their learning enthusiasm.

#### 4.1.1. Create an Excellent Classroom Teaching Environment

The education of ecological civilization is an important subject closely related to human living environment [18]. This is closely related to building a better China and a civilized ecological society, as shown in Tables 2 and 3. Universities are the main body of ecological civilization construction. At present, the overall level of college English classroom teaching environment in China is low, and students' learning enthusiasm is not high. Creating a good learning atmosphere is conducive to cultivating students' ecological consciousness. In order to cultivate students' subjectivity and initiative, we need to create a good classroom atmosphere through various ways. On the one hand, the state has issued a series of laws and regulations to protect the ecological environment and provide institutional guarantee for creating the classroom teaching environment. On the other hand, a publicity and education system led by the government, coordinated by official associations and individuals, has been formed to improve the enthusiasm and initiative of university students in protecting ecological civilization, from unidirectional to multidirectional expansion, forming a multidirectional joint force of various departments.

#### 4.1.2. Strengthen the Construction of School Spirit and Study Spirit in Ecological Education for College Students

In order to realize ecological protection, in addition to establishing a good campus cultural atmosphere, there should be corresponding policies and severe punishment for the behavior of destroying the ecology. The school spirit, class spirit, and study spirit of colleges and universities are invisible systems, which profoundly affect the thought, behavior, and consciousness of college students as well as their ecological consciousness, thus enhancing the effectiveness and effectiveness of ecological education of college students. Colleges and universities should construct the ecological construction system which is suitable for the ecological practice of college students and strengthen the restriction between the education subject and the educatees, so as to form the resultant force of ecological protection and enhance the consciousness and consciousness of college students. Campus culture is a kind of spiritual outlook and the most precious spiritual wealth of colleges and universities [19]. Class style is a kind of learning habit and behavior formed in the class collective; this habit will have a certain influence on students' learning enthusiasm and initiative and then have a certain influence on their future. Class style is a class to develop a learning habit and behavior; it may affect their enthusiasm and initiative, so as to affect their future, so as to affect their growth. To strengthen the construction of ecological civilization in colleges and universities, we must establish good school spirit, class spirit, and study spirit. To strengthen the construction of the style of study, we should start with correct students' learning attitude and guide them to establish a correct concept of interests (see Figure 7).

### 4.2. The Optimization Strategy of Ideological Education of College Students in the New Era

The ecological problems of ideological and political education of college students in the new era have both internal and external causes [20]. College students' ideological and political education activities should give full play to the role of various factors on the basis of following the ecological law, adhering to the basic principles of comprehensive, being integral, coordinated, and sustainable, and strengthening the interaction of information and energy transmission. We explore from the following aspects.

#### 4.2.1. Change Subject Cognition to Enhance Overall Awareness

The development practice is based on a certain development concept, and the correctness of the positioning concept directly affects the effect of the practice. In order to meet the needs of the new situation and the new period, we must thoroughly change the traditional way of thinking from the understanding and reality, so that the ecological idea of ideological education can be truly carried out in the whole teaching activities. Cultivate ideological education subject.

- The concept of “big ideological and political” mode is closely combined with the needs of the overall ideological education. It is necessary to comprehensively grasp and design at the top level the ideological and moral construction of students and solve the problem of unbalanced and inadequate development in a targeted way, so as to meet the requirements of the development of students' ideological education in the new era. We should attach great importance to the integration of education and teachers; strengthen exchanges and interactions from the party committee, student work, department leadership, subject teachers, counselors, and other aspects; do a good job of linking up, forming complementary advantages of the work situation; and really give full play to the strengths and characteristics of full-staff education
- To understand the ecological orientation of ecological subject scientifically is to correctly understand its role in education and teaching activities, so as to keep its dynamic balance in the new era

#### 4.2.2. Deepen Theoretical Research to Enhance Theoretical Confidence

Only by fully affirming and trusting it, can it be better materialized into practice, and only by fully affirming and trusting the theory of state can ideological and political educators better materialize into practice and consciously realize the unity of theoretical logic and practical logic. To do a good job of ideological education in colleges and universities and strengthen theoretical research is directly related to the identity and belonging of the subject but also related to the validity and initiative of ideological education subjects to use theoretical knowledge to guide and improve educational problems.

#### 4.2.3. Integrate Various Resources to Enhance the Resultant Force of Education

They are closely related to family education. To strengthen school education, one should establish a scientific and harmonious concept of family education, parents should take the way of education should be combined with the actual situation of children, starting from reality, reasonably learn from the education theory of education experts, really from the heart of children, concerned about their psychological development and ups and downs. The second is to strengthen the thought and guidance of family education. For scholars, the head of the family is more of a role of moral education and wisdom in life. Parents should guide the direction of ideological understanding, develop the influence and influence of parents, and create a warm education environment for scholars. The parents keep in touch and communicate with the school. Great scholars are the backbone of family education, and their educational practice can really solve their thinking problems of embodied reality. Home education is not only to improve the effect of ideological and political education but also to help scholars become talents, to benefit the infiltration of ideological and political education, so that ideological and political education can play a long-term role.

## 5. Conclusions

The ideological education ecosystem for college students is a complete system of interdependence and mutual openness. In the long process of development, each factor can form a harmonious, balanced, and complementary relationship and create a harmonious and stable social environment for the comprehensive and free development of people, thereby improving the teaching efficiency of the school. The thoughts and values of college students are important factors influencing social values. On the basis of adhering to being “people-oriented,” we should strengthen the moral guidance of the ideological education of college students and establish and improve the ideological education system for college students. This paper mainly studies the basic issues of student ecological education, including the concept, content, and significance of student ecological education; problems and causes of student ecological education; and ways to solve problems in student ecological education.

## Figures and Tables

**Figure 1:** Classroom ecological structure diagram.

**Figure 2:** The importance of ecological civilization education in colleges and universities.

**Figure 3:** Schematic diagram of school cultural ecosystem.

**Figure 4:** Teaching methods of ecological civilization.

**Figure 5:** Emphasis on ecological civilization literacy.

**Figure 6:** Support for national ecological civilization construction.

**Figure 7:** Schematic diagram of the main contents of efficient ecological civilization education.

**Table 1:** Ecological knowledge mastery table.

The title	Correct
What was the first international conference where the world's governments discussed contemporary environmental issues and discussed strategies to protect the global environment?	29.69%
Which day is Earth Day, one of the three major environmental holidays?	53.85%

**Table 2:** Set up ecological civilization education courses.

Options	Students	Accounted for
Have the necessity of opening	207	42.00%
Do not know	128	26.00%
It is not necessary	98	20.00%
Other	59	12.00%

**Table 3:** Whether the school offers ecological civilization education courses.

Options	Students	Accounted for
Has a set-up	130	26.50%
Did not open	263	53.50%
Do not know	98	20.00%

## Data Availability

The labeled data set used to support the findings of this study is available from the corresponding author upon request.
